# Virtual Reality Technology of New Media Visual Simulation

This article has been retracted.

**DOI:** 10.1155/2022/8978152

**Published:** 2022-08-25

**Authors:** Feng Li

**Affiliations:** School of Humanities and Arts, Nanchang Institute of Technology, Nanchang, Jiangxi, China

## Abstract

In order to improve the exhibition effect of museums and expand the display ways of digital museums, a Chinese museum scene roaming application system based on the Unity 3D virtual reality engine was proposed. 3Dmax model production software was used to complete the museum scenes and the model production, material, and lighting of collections in the museum. Through the Unity 3D virtual reality engine, the design and production of the interactive system were completed. The display and application of the scene roaming system of the Chinese museum were well realized. For the system, the fast construction of virtual scenes and fixed-point triggering (FPT) optimization were carried out. The experimental results showed that the improved method was 90.5% faster than the manual coding method in the optimization of fast virtual scene construction. After using the fixed-point triggering method, the average accuracy of the original 35 scenes was 63.9%. It was concluded that the application design could simulate the museum scene well, which had a certain reference value for the application of virtual reality simulation technology in the field of cultural heritage inheritance.

## 1. Introduction

This way of conveying information is passive, monotonous, and boring to the audience, which cannot reproduce the exhibits completely and lacks the expressive force [1, 2]. The most fresh force of new media art for display design is to rely on its high-tech media technology, which changes the display carrier from material to nonmaterial and changes the display form from static to multidimensional dynamic display at the same time, realizing people's more diverse, novel, and unique needs for art. In the age of new media art, the old physical display has been replaced by 3D virtual imaging technology, which allows many unreproducible objects and things that do not exist to be presented. At the same time, it can produce different spatial forms within a limited area, which greatly saves space, materials, transportation, and other material resources. So, it enables people to get a variety of sensory experiences in a small place [3].

On the basis of this research, this paper proposes a new media visual simulation and virtual reality technology research. The application design can simulate the museum scene well and has a certain reference value for the application of virtual reality simulation technology in the field of cultural heritage inheritance.

This paper uses 3Dmax model making software to complete the production of museum venues and collections in the museum, then exports it to FBX format and imports it into Unity3D software, uses C# script to complete the interactive action design, and finally packs the completed project into an APK file and exports it to VR hardware used in. The VR hardware used in this project is the Samsung S6 mobile phone, and the S6 is inserted into the Gear VR glasses, and the virtual roaming and interaction of the Chinese museum can be completed only by wearing the VR hardware. Using virtual reality technology, we can convey the stories, culture, and other content behind the cultural relics to people, just like leading people to travel through history.

## 2. Literature Review

Since the beginning of the 21st century, digitalization, integration, networking, and intelligence have had a significant impact on the development of museum exhibitions. Therefore, countries with relatively developed digital technology and culture attach great importance to the digital development of museum exhibitions. Bran developed an augmented reality museum guide system based on mobile terminals. The system could not only provide information about the exhibits' internal structure, relevant origin information, and usage method but also interact with exhibits. The mobile terminal system used in this system was the ultramobile personal computer (UMPC), which integrated cameras, ultrasonic receivers, gyro sensors, and other devices [4]. Schuster took a national museum as an example to investigate the effect of AR (augmented reality) technology on the learning effect of cultural relics visiting experience in an informal learning environment through a large-scale field experiment. Experimental results showed that exhibits based on AR technology not only had high value but were also very popular in museum exhibitions [5]. Manca adopted the experimental research method to compare AR museum guides and audio guides with nonuse guides. The influence of different guidance systems on users' art appreciation was evaluated through pre and posttests with the same content [6]. Torres-Ruiz took small and medium-sized museums in a city as an example to point out the current situation that small and medium-sized museums have a single way of displaying cultural relics. They proposed that augmented reality technology could solve the problem of small and medium-sized museums having a single way of displaying cultural relics and a lack of interactive experience. It is also pointed out that the construction of development applications based on mobile platforms and augmented reality technology had certain practical significance in improving the experience of visitors [7]. Khan summarized the artistic features and advantages of augmented reality technology in museum display by analyzing excellent cabinets of augmented reality at home and abroad [8].

In the research, 3Dmax model production software was used to complete the production of museum scenes and collections in the museum. Then, it was exported to FBX format and imported into Unity3D. C# script was used to complete the interactive action design. Finally, the completed project was packaged as an APK file and exported to VR hardware for use. The VR hardware used in the research was a Samsung S6 mobile phone, and the S6 was inserted into the Gear VR glasses. The virtual tour and interaction of the Chinese museum could be completed only by wearing VR hardware. It was noted that the system implementation in the research was based on Gear VR hardware, so part of the system code involved in this platform was called from the Gear SDK and only applied to the Gear VR hardware. In this study, the virtual roaming display of the museum is well realized, and the human-computer interaction action event design is added in the roaming process. To improve people's interest in learning and visiting and to perceive the charm of Chinese cultural relics in an “immersive” way, at the same time, applying virtual reality technology to the reproduction technology of museums is also a feasible way to explore the field of cultural heritage protection.

## 3. Research Methods

### 3.1. Overall Design

#### 3.1.1. Tools and Methods

In the research, Unity 3D is used as a system development tool. 3Dmax is used as the model production tool and the materials and lighting are provided. The 3D model of the completed scene and exhibits is exported to the FBX file format and imported into the Unity 3D project file. C# is used as the scripting language to achieve the virtual interactive system design of the museum scene. Through the materials and lighting, the effects of real exhibits are simulated. In particular, the research focuses on experimental research on system design, so a lot of model simulation is not done in the process of model building [9]. The real museum scenes and exhibits are extremely rich, but the research does not make in-depth discussion.

#### 3.1.2. Interaction Design

After the scene construction of the platform is completed, interaction design needs to be completed in Unity 3D. Human-computer interaction is set for action in Exhibition Hall 2. The Gear touchpad can be used to select exhibits [10, 11], which can be rotated and zoomed in and out. The venue plan is shown in Figure 1.

The specific path set by this platform (Figure 2) is that when entering the scene, the “centering focus” museum plaque is first set and the plaque flashes at the same time. When the “centering focus” is completed, the plaque no longer flashes. The museum text introduction appears immediately below the plaque. After a period of time, the text disappears, and the camera moves, and the camera passes through Exhibition Hall 1 and Exhibition Hall 2. Visitors (players) can move and rotate to visit the exhibits on the walls of the exhibition hall. Visitors decide the visit time in Exhibition Hall 3 or Exhibition Hall 4. When visiting is finished, visitors arrive in the middle position (position) of Exhibition Hall 3 or Exhibition Hall 4. The camera begins “centering focus” on an exhibit when the glass outer frame of the exhibits stops flashing [12].

### 3.2. System Implementation

#### 3.2.1. “Centering Focus”

When visitors enter the virtual museum display platform, the screen starts to move as follows. “Centering focus” focuses on the China museum plaque, the plaque which flashes. When the reading of the progress bar is finished, the plaque is no longer flashed. The plaque effects show white text on the “Chinese Museums are the main collection of specimens of Chinese cultural relics and institutions, publicity and education institutions, and scientific research institutions, which is an important part of Chinese socialist scientific and cultural undertakings.” After a period of time, the words disappear [13]. The specific process is given.

(1) The crosshair progress bar reading: The camera (len) is equivalent to ray and ray is our line of sight, which is called from the Gear SDK. When we look at the object, the crosshair progress read animation is triggered. The schedule loading animation lasts for about 3 s or so and then triggers the other logic (plaque flashing).

(2) Plaque flashing: In order to make the effect of plaque flashing look more realistic, the frequency of plaque flashing is set as random in this system, and the interval between the beginning and end of each flash is taken according to the time parameter given by the system. This design avoids the overly mechanical effect of the plaque flashing, which is also consistent with the real-light flashing effect. The specific design process is shown in Figure 3.

(3) Text introduction: When the centering progress bar is read and the plaque stops flashing, the museum text introduction will appear immediately. After a while, the text fades out until it disappears. The length of the text introduction is set according to people's normal reading speed (the average reading speed of ordinary people is 300–500 words/min). The length of text display on this platform is 6 s. When the text disappears, it goes to the next logic.

#### 3.2.2. Display Cabinet Frame Flashing

In order to attract the attention of visitors, the system platform sets the flashing effect on the glass display cabinets of all exhibits in Exhibition Hall 2. When visitors enter the scene, the glass frame immediately starts flashing. When the person moves to the display cabinet of the exhibit and wants to visit the exhibit, he can stare at the corresponding exhibit for a few seconds. At this moment, the outer frame of the glass display cabinet stops flashing and the centering progress bar starts to load at the same time. When the loading is completed, the exhibit moves to the eyes of the visitor (Gear VR hardware wearer). The code of “Player moves” is that when the visitor (player) reaches the designated position in Exhibition Hall 2, the glass frames of all exhibits are flashing [14]. At this moment, the visitor can “focus” on any glass cabinet. When the progress bar “centering focus” starts to load, the glass frame stops flashing. Exhibits in glass frames move to the front [15]. The specific design process is shown in Figure 4.

The system code of “flashing” is attached to the glass frame. The effect is that when the glass frame starts flashing, it flashes at a rate of once per frame. The process is as follows.

1. First, the previous script “Player moves” is mounted to the camera. Once it starts running, the code is executed in a loop within a fixed time to record the camera position. When the camera position value is within a certain value, the next logic will be triggered.
2. The “flashing” script is mounted to the glass outer frame, and the current logic will run properly to trigger this logic. If the previous logic does not run, it will not trigger this logic.

#### 3.2.3. Change of Physical Properties of Relevant Objects and Realization of Triggering Events

In the roaming process of the platform, the Gear VR trackpad can be used for interaction in some areas. The system code for using the touchpad is called from the Gear SDK.

#### 3.2.4. Design of Character Movement, Explicit, and Implicit Events

In the running process, there is a script that is most frequently used, temporarily named as “Scripts.” It involves the character's movement, objects visible and hidden, objects reset, rotation reset, zoom in and zoom out, and reset. The specific approach is to complete the logical connection according to the real-time position and focusing parameters of Gear VR (Unity 3D is seamlessly connected with Gear VR and parameters are assigned to the machine according to the position and focusing properties of the wearer) [16], as shown in Figure 5.

#### 3.2.5. Exiting from the Exhibition

The exit method designed in the research is that “centering focus” focuses on an object, and the exhibition is exited after about 2 s. The specific idea is that when we have visited all the exhibits in Exhibition Hall 2, we return to the designated position and “centering focus” again on the wooden box in the museum. The camera starts to move and finally returns to the position at the beginning of the platform. Visitors can choose to visit again or end the visit. The above implementation code technology is basically consistent with the interaction settings after the platform enters the market, so the technical ideas will not be described here. Considering that after the current visitor finishes the visit, the next visitor can enter the visit directly and quickly, an overly complicated interactive mode in the setting of the ending effect is not chosen.

### 3.3. Improved Methods for Rapid Construction of Virtual Scenes

A coded build method is often used when loading large numbers of data objects or models into a normal area of a virtual scene. However, the traditional method is not suitable for constructing models in irregular scene areas. In the construction of a scene model in an irregular scene area, it is necessary to manually modify or move the direction and size of each object or model, which requires a lot of time and energy and will inevitably affect the time cost of the construction of the whole virtual scene [17]. Therefore, the coded build method is not suitable for batch loading models in irregular scene areas. Therefore, in the research, the spline curve method is used to determine the model placement points in the irregular scene area.

### 3.4. Fixed-Point Triggering (FPT) Method

In the scene production of the virtual museum tour, due to the requirement of scene authenticity, all models are completed with high precision. High-precision 3D models such as walls, war drums, murals, porcelain, bronzes, and display cabinets will lead to a declining running frame rate of the whole platform [18]. In order to solve this problem, a fixed-point triggering (FPT) method is proposed based on the combination of a simple grid and an iTweenPath plug-in in the research. The specific steps of the method [19] are as follows.

1. Use simple grid plug-in and detail level (LOD) technology to reduce the triangles on the model surface for rendering, improve the frame rate of part of the platform operation, and merge the 3D model grid with the rendering mode set in the 3D scene.
2. Use the visual editing path function of the iTweenPath plug-in to complete the setting of the camera roaming path in the virtual scene according to the specified roaming route
3. Set appropriate subtitles and voice triggers on some fixed points of the roaming path of the scene
4. If the camera does not roam to the last control point, step (5) is entered. Otherwise, the roaming process is ended.
5. When the camera roams to the corresponding trigger point, the corresponding subtitles and voice are triggered until the end of roaming

## 4. Result Analysis

### 4.1. Experiment Effect Analysis of the Improved Method for Rapid Construction of Virtual Scenes

Scenes I–VI are, respectively, captured in the virtual museum's roaming system. The traditional manual coding method and the improved method are, respectively, used to construct the scenes, such as the way the model is built and the time to run the program. The time cost is shown in Figure 6.

The time cost in Figure 6 is the average of the experiments. Data comparison shows that the improved method is 90.5% faster than the manual encoding method on average. When models are loaded in batches in conventional or irregular scene areas, the time cost of the improved method of virtual scene construction proposed in the research is far less than that of the traditional manual coding method, which can save a lot of time. The model location is more accurate.

### 4.2. Analysis of Experiment Effect of the Fixed-Point Triggering (FPT) Method

In the fixed-point triggering experiment, all scenes in the platform are recorded and tested manually. The virtual scenes of 35 museums are designed in this virtual museum tour design. In the results of experimental analysis, if the time difference between each subtitle, voice, and scene is within 2/3 seconds, the record is marked as a match. Otherwise, the record is marked as a mismatch. The matching rate of a scene is the average accuracy rate of the scene, as shown in the following formula [20].

(1) $$\begin{array}{c} \text{MAP}=\frac{\sum_{i=1}^{n}T_{i}/T_{i}+F_{i}}{n}. \end{array}$$

In formula (1), *n* represents the number of virtual scenes, *T*_*i*_ represents the number of matching records in the *i*th scene, and *F*_*i*_ represents the number of mismatching records in the *i*th scene. Finally, the proposed average accuracy evaluation criteria listed in formula (1) are used to calculate the average accuracy of 35 scenes [21, 22].

Experiment results show that the average accuracy of the original 35 scenes is 63.9%. After adopting this method, subtitles, speech, and scenes can always match each other [23–25].

## 5. Conclusions

In the research, the virtual roaming display of the museum was well realized. At the same time, human-computer interaction in the process of roaming action event design was added. By operating the virtual reality peripheral equipment, the museum of the scene could be displayed and the man-machine interactive experience could be completed, which raised people's interest in learning to visit. The charm of Chinese cultural relics could be felt in the form of “immersive.” At the same time, applying virtual reality technology to the reproduction technology of museums could be regarded as a feasible way to explore the field of cultural heritage protection. The specific conclusions are as follows.

1. Ancient cultural relics are protected in the museum. In order to protect ancient cultural relics from damage, they are collected in the exhibition cabinet. Due to the distance limitation of the exhibition cabinet, visitors cannot see the details of the exhibition objects at a close distance nor can they see the partially blocked by the exhibition cabinet. Virtual technology helps museums solve this problem by putting cultural relics in the virtual environment and presenting them realistically in front of people, which also ensures that cultural relics are not damaged.
2. Museums are full of profound cultural connotations. Culture is the historical culture from ancient times as contained in ancient books of cultural relics. Virtual reality technology can convey the stories and culture behind cultural relics to people, just like leading people to travel through history.
3. Virtual restoration of cultural relics and data storage are sustainable in the museum. Even if the cultural relics are protected in various ways, embrittlement, decoloring, and peeling still appear. Virtual reality technology can be used to display, protect, and repair cultural relics. At the same time, all of the cultural relics can be stored in the database forever.

Through the design and application of this platform, we found that Unity 3D supports almost all custom materials and can call and manage models, materials, lights, and even animations in the form of scripts. The application design can simulate the museum scene well. The application of virtual reality simulation technology in the field of cultural heritage inheritance has a certain reference value. In addition, the seamless connection between Unity3D and Samsung Gear VR, HTC VIVE, and other virtual reality somatosensory devices provides more ideas for the design of this system platform and the design practice of many similar platforms.

## Figures and Tables

**Figure 1:** Plan of the museum.

**Figure 2:** Operation diagram of museum roaming platform.

**Figure 3:** Flowchart of the plaque flashing system.

**Figure 4:** Design of the glass outer frame flashing system.

**Figure 5:** Schematic diagram of logic connection.

**Figure 6:** Comparison of experiment time cost between the two methods.

## Data Availability

The data used to support the findings of this study are available from the corresponding author upon request.
